The article "Development of the 8-Item Phlegm Pattern Questionnaire (PPQ-8) Using Rasch Analysis" was published in 2021. Journal: Evid Based Complement Alternat Med.

# Development of the 8-Item Phlegm Pattern Questionnaire (PPQ-8) Using Rasch Analysis

**DOI:** 10.1155/2021/6528891

**Published:** 2021-10-28

**Authors:** Young-Jae Park

**Affiliations:** ^1^Department of Biofunctional Medicine and Diagnostics, College of Korean Medicine, Kyung Hee University, 26 Kyungheedae-ro, Dongdaemun-gu, Seoul 02447, Republic of Korea; ^2^Department of Diagnosis and Biofunctional Medicine, Kyung Hee University Hospital at Gangdong, No. 892 Dongnam-ro, Gangdong-Gu, Seoul 05278, Republic of Korea

## Abstract

The 25-item Phlegm Pattern Questionnaire (PPQ) has been widely used to examine the relationship between the phlegm pattern (PP), quality of life, tongue colour, vocal qualities, and dysfunctional breathing. However, the concerns of response burden and differences in the respondent's abilities or item difficulty for the original version of the PPQ have not been sufficiently addressed. This study aimed to develop a short-form PPQ using Rasch analysis, an item response theory. Based on the retrospective data, the response order, differential item functioning (DIF), dimensionality, reliability, concurrent validity, and fitting errors were examined for 291 normal participants and 61 inpatients. The discriminative ability of the short-form PPQ was examined using receiver operating characteristic curve analysis. Along with Rasch analysis, another short-form PPQ was developed using equidiscriminative item-total correlation (EITC) analysis and the results between the two short-form PPQs were compared accordingly. Rasch analysis results suggested a 6-point response category for the PPQ, and finally, 8 items without fitting errors or DIF variability were selected for the PPQ (PPQ-8). The PPQ-8 had satisfactory reliability (person separation index = 2.23), unidimensionality (unexplained variance in the first contrast = 1.598), fitting levels (infit mean square, 0.80–1.39; outfit mean square, 0.79–1.34), sensitivity (70.5%), and specificity (76.5%). The PPQ-8 had a moderate discriminative ability of the PP (area under the curve = 0.759), and the cut-off point was 23. Although the 8-item PPQ developed using EITC analysis showed similar levels of reliability, validity, and discriminative ability of the PP to the PPQ-8, it could not present the information of item hierarchy and differences in the respondents' abilities. In conclusion, the PPQ-8 by Rasch analysis is recommended for future use to evaluate the clinical severity of PP.

## 1. Introduction

According to the traditional Chinese medicine theory, a pathological pattern is a subcategory of a disease or disorder referring to a diagnostic conclusion based on the pathological changes at a certain stage of disease [1]. Pathological patterns are efficient in population health management [2, 3] and can be applied to guide the prevention, treatment, and rehabilitation of diseases [4]. Among the diverse pathological patterns, phlegm is a viscous, turbid pathological product that accumulates in the body and covers the areas where fluid or lymphatic circulation may be retarded [5]. Similar to traditional Chinese medicine, Korean medicine recognises that the accumulation of phlegm leads to nasal discharge or sputum and diverse neurological and gastrointestinal problems, including dizziness, palpitation, ingestion, and mucousy stool [6]. Interestingly, traditional Persian medicine has recognised that the balance among the “4 humours” (black bile, yellow bile, phlegm, and blood) in the human body sustains health preservation, while the lack of this balance results in diseases, especially the dystemperament state [7]. The presence of phlegm in the body can be diagnosed by examining the signs and symptoms in the patient's clinical history [8]. Due to the wide spectrum of pathophysiology and high affinity towards other pathogenic factors, a Korean medical doctor must identify the presence of phlegm. A phlegm pattern (PP) is a pathological condition caused by phlegm [8]. A Phlegm Pattern Questionnaire (PPQ) was developed to quantitatively evaluate the clinical severity of PP [6]. A self-administered PPQ consists of 25 items, with each item rated on a 7-point Likert scale (1 = disagree very strongly and 7 = agree very strongly).

The PPQ was reported to have satisfactory reliability (Cronbach's alpha coefficient = 0.902) and the moderate discriminative ability for PP (area under the curve (AUC) = 0.860) [6]. Since its development, PPQ has been utilised to evaluate the clinical severity of phlegm in diverse physiological or pathological conditions in the body. For example, increased clinical severity of PP, estimated by the PPQ scores, was associated with other pathological patterns, including increased clinical severity of yin deficiency manifesting with emaciation, tidal fever, night sweats, and increased clinical severity of qi deficiency manifesting as fatigue, shortness of breath, and indigestion [8], thereby causing a decline in the quality of life [9]. In a study on the relationship between quantitative tongue colour and pathological patterns, decreased yellow colour of the tongue tip was related to increased PPQ scores [10]. Furthermore, the vocal quality of normal subjects, especially decreased tremor-related parameters and increased resonance-related parameters, was found to be associated with increased PPQ scores [11]. Recently, a study reported higher PPQ scores in a dysfunctional breathing group than in a nondysfunctional breathing group, suggesting that the clinical severity of phlegm may be associated with the aggravation of dysfunctional breathing [12].

The length of the original version of a questionnaire often limits the extent to which it applies to patient care or research [13]. A large number of questionnaire items require excessive time for completion; in particular, the questionnaire length or the multipurpose battery of different questionnaires can affect patients with difficulty in handwriting or cognition [13]. Therefore, a demand to reduce the burden of response and a few methodologies to reduce the questionnaire items previously developed have been raised in the past. For example, Beaton et al. shortened the original version of the 30-item Disabilities of the Arm, Shoulder, and Hand Outcome Measure (DASH) and developed an 11-item QuickDASH [14]. Similarly, Badia et al. developed a 16-item Osteoporosis-Specific Quality of Life Questionnaire [15]. Furthermore, Kim suggested reducing the short-form health survey questionnaire (SF-36) to an 11-item questionnaire [16]. However, no study has addressed the item reduction of the 25-item PPQ. Therefore, this study aimed to develop a short form of the PPQ to reduce response burdens, such as answering time or difficulty in handwriting or cognition. One of the conventional statistical methods to reduce questionnaire items is to examine item-total correlations (ITCs) for each item [17]. Using ITCs, the top-ranked items can be retained, while lower-ranked items may be deleted accordingly. The equidiscriminative item-total correlations (EITCs) constitute a modified ITC method in which ITC analysis is repeated three times based on low, medium, and high score points. EITC has the advantage of distinguishing between respondents throughout the range of the total scores [14, 18]. However, the classical methodology has the limitation of not considering item hierarchy, that is, the characteristics of item response. Rasch analysis is an item response theory where each item response in the questionnaire is taken as an outcome of the independent interaction between the respondents' abilities and item difficulty [19]. If the item the weightings are ordered based on their difficulty along a linear logistic function, multiple response options, that is, the Likert scale, may be acceptable [14]. Through the examination of response difficulty, the overlapping response category may be deleted or unified suitably, and the number of response categories can thus be reduced. Rasch analysis presents information on whether each item fits a linear function. Misfitting items derived from an acceptable fit level may be removed from the questionnaire [13]. Moreover, Rasch analysis presents the data of differential item functioning (DIF), which identifies items that do not function equally among different groups of respondents [20]. Through the DIF process, a questionnaire with reduced items may become robust, irrespective of group differences, such as gender or age. In summary, this study aimed to develop a short form of PPQ following EITC and Rasch analyses and to examine the discriminative power of PP using receiver operating characteristic (ROC) curve analysis.

## 2. Methods

### 2.1. Data Sources

The data used for analysis in this study were collected for the development of the PPQ [4]. The 25-item PPQ is shown in Table 1. The data used to develop the original version were completed by 291 normal participants consisting of 132 men (mean age, 39.81 ± 19.39 years) and 159 women (mean age, 43.61 ± 15.21 years), who consulted a clinician for a health consultation [6]. In a previous study [6], three clinicians blindly determined the presence or absence of PP in 61 inpatients, where they investigated the same patients successively at 10 minute intervals to minimise the interobserver variability, and the results of their decisions remained blinded. The final determination of PP was accepted only when at least two clinicians diagnosed an inpatient with PP. The PP data from the previous study were used to examine the discriminative ability of the short-form PPQ in this study through ROC curve analysis. To compare the internal consistency, validity, and discriminant power of the short-form questionnaire with the original version of the PPQ, the data of normal participants and inpatient groups in this study were considered equal to those of normal participants and inpatient groups in the previous study. The study protocol was approved by the Institutional Review Board of the Kyung Hee University Oriental Medical Hospital at Gangdong (IRB approval number: KHNMCOH 2021-02-001).

### 2.2. Rasch Analysis

A conventional questionnaire development assumes equal weighting for each item and uniform intervals between the responses for each item. However, these assumptions may not be true as the difficulty of items and the ability of the subjects to answer an item often vary. Therefore, in this study, the first step of Rasch analysis was to evaluate the weighting and difficulty of each item and rescale the 7-points Likert scale of the PPQ if there was any disordering of item responses. In the next step, the DIF, which emerges when the responses to an item function equally in different subgroups of participants for the 25-item PPQ, was evaluated. In most cases, external factors, including age and gender differences, result in DIF, and items affected by DIF would be deleted from the original version of the questionnaire [20, 21]. Rasch modelling assumes that items are weighted according to their difficulty along a linear logistic function. The mean square error (MnSq) is the chi-square statistic divided by the degrees of freedom [13]. If an item fits this linear function, the MnSq of the item ranges between 0.5 and 1.49 [22]. Therefore, in the third step of this modelling, the MnSq levels of the two fit indices, infit and outfit, were evaluated. Misfitting items were deleted, and iterations of fit evaluations were conducted until only fitting items remained [14]. Finally, the reduced items were checked for additional dimensionality. The determination of unidimensionality helped avoid scoring unrelated dimensions within the reduced items.

### 2.3. Equidiscriminative Item-Total Correlations

EITC, a modified ITC, is used for item reduction in a questionnaire [23]. While ITC focuses on the correlations between the scores of each item and the total scores of a questionnaire, EITC resets three cut-off points according to the three percentile levels of the total scores (25%, 50%, and 75%) and transforms the total scores for each individual into dichotomous values [18]. In this study, the values below and above the cut-off points of 25% were transformed to scores of 0 and 1, respectively, and dichotomous total scores were assigned to all participants. Similarly, other dichotomous total scores were determined according to cut-off points of 50% and 75%, respectively. Thereafter, correlations between the three sets of dichotomous value-transformed total scores and questionnaire item scores were examined, and the EITC for each item and the dichotomous value-transformed total scores were sequentially ranked according to the three percentile points. The weights of EITC did not differ between each percentile group, and items with the highest values were extracted from each subgroup by multiples of three. Therefore, the top three or four items were sequentially collected in the order of 25%, 50%, and 75% EITCs, and a total of 9 or 12 items were preliminarily determined as a short-form questionnaire [14]. If the same item was in the top four lists for both the 25% and 50% categories, it was dropped from the list of the 50% group, and the next ranked item from that group was substituted into the 50% list. Similarly, the item in the 75% list was dropped, and the next ranked item was substituted if it was both in the 50% and 75% ranks [14, 18]. The final determination of the item numbers obtained using EITC was matched with those obtained using Rasch analysis, according to a previous study [14].

### 2.4. Receiver Operating Characteristic Curve Analysis

A previous study defined an optimum cut-off point of 5 points on the 25-item PPQ and reported the AUC level of the PPQ, which is a discriminative PPQ power [6]. In this study, sensitivity, specificity, AUC levels, and cut-off points of the short-form questionnaire developed by EITC and Rasch analysis were calculated accordingly. Discriminative powers of the two short-form questionnaires were then separately compared with those of the 25-item PPQ.

## 3. Statistical Analysis

### 3.1. Rasch Analysis

Rasch analysis was conducted using the partial credit model as each item was answered in the form of a polytomous category, that is, a 7-point Likert scale [19]. The ordering of the item response was acceptable when the following conditions were satisfied: (1) total counting numbers of each response category ≥10, (2) ascending ordering of average measure and step calibration, and (3) outfit level of each category ≤2.0 [24]. If there was any violation among the item response category, the category was unified with an adjacent category, and the ordering of all categories was re-evaluated. Along with the numerical examination, the category probability curve was extracted and examined for the overlapping of a category curve peak with other curves [25]. An overlapped curve indicates a disordering of the response category. DIF was assessed for both sex and age. The median age of the participants was 46.0 years, and those over and below 46 years were assigned to the older and younger groups, respectively. Differences in logits between men and women and the older and younger groups were examined using the chi-square test and *P*-values. Infit and outfit were assessed, and items with MnSq infit or outfit values <0.50 or >1.50 were removed, respectively [22]. Similar to ETIC, the dimensionality of the reduced items was assessed by principal component analysis. In Rasch analysis, unidimensionality was determined when the unexplained variance in the first contrast was under 2.0, where the number of the second factor may have consisted of only one item [26]. Reliability was examined using a person separation index, where values ≥ 2.0 were considered “acceptable” [27].

### 3.2. Equidiscriminative Item-Total Correlations

EITCs were calculated using Spearman's rho correlation because of the dichotomous values for the total scores. The dimensionality of the reduced items was assessed using principal component analysis. In the EITC, the number of dimensions was examined with an eigenvalue of over 1 point. The concurrent validity of the two short-form questionnaires was examined using Pearson's correlations between the total scores of the original version and the short-form PPQ by EITC. Internal consistency was examined using Cronbach's alpha coefficient with values of ≥0.9, 0.7–0.9, and 0.6–0.7, which were considered excellent, good, and acceptable, respectively [28].

### 3.3. Receiver Operating Characteristic Curve Analyses

After examining the reliability, validity, and dimensionality of the two short-form questionnaires, ROC curve analyses of the EITC and Rasch modelling were conducted, where the total scores of the reduced EITC and Rasch items served as test variables, and the presence or absence of the PP, identified by three clinicians, served as a gold standard. The discriminative ability of the reduced questionnaire was evaluated using the AUC. As generally accepted, AUC with values > 0.9, 0.7–0.9, and 0.5–0.7 indicated high, moderate, and low accuracies, respectively [29]. An optimum cut-off point, the Youden index, was examined using two statistical values (Youden index = sensitivity + specificity – 1) [30] and the Euclidean distance from the left-top angle to the ROC curve, where the *x*-axis represents the 1-specificity value and the *y*-axis represents the sensitivity value (Euclidean distance = $\sqrt{{\left(1-\text{sensitivity}\right)}^{2}+{\left(1-\text{specificity}\right)}^{2}}$) [31]. An optimum cut-off point corresponded to either the maximum Youden index or the minimum Euclidean distance. EITC and ROC curve analyses were performed using SPSS version 21 (IBM Corp., Armonk, NY, USA), and Rasch analysis was performed using Winsteps 4.8. Statistical significance was set at *P* < 0.05.

## 4. Results

The category characteristics of the 25-item PPQ are summarised in Table 2. The original version of the PPQ was rated on a 7-point Likert scale (1 = disagree very strongly; 2 = disagree strongly; 3 = disagree; 4 = neither disagree nor agree; 5 = agree; 6 = agree strongly; 7 = agree very strongly), and whether the 7-point category responses were in an increasing order was examined accordingly. The total counting numbers of each category exceeded 10, and their outfit MnSq levels were below 2.0. However, the step calibration or threshold scale for category 4 (“neither agree nor disagree”) decreased more than that of category 3 (“disagree”), indicating that both categories 3 and 4 were disordered among the category responses.  Figure 1(a) shows the probability curve of question 1 (“I have a cough”), according to the 7-point Likert scale, where the peak of category 3 overlapped with that of category 4, consistent with the results of step calibration. This peak overlapping of category 3 with category 4 for question 1 was similarly found for the other 24 question items. Therefore, categories 3 and 4 were unified, and a 6-point Likert scale was used for the Rasch analysis. The step calibration of the 6-point categories maintained an increasing order (Table 2).  Figure 1(b) shows that the category curves were ordered correctly without overlapping of the peaks, although the peak of category 4 was barely exposed.

Table 3 lists the DIF results according to gender and age. The logit values for “cough (Q1),” “sputum (Q2),” “abdominal rumbling (Q8),” “mucousy stool (Q17),” and “itching (Q24)” in men were higher than those in women, while the logit values for “palpitation (Q14),” “startled by faint noise (Q15),” “joint pain (Q19),” “limb heaviness (Q20),” and “yellow face (Q23)” in women were higher than those in men. In age groups, the logit values for “sputum (Q2),” “feeling of foreign body (Q3),” “abdominal rumbling (Q8),” “sickness (Q9),” “headache (Q11),” and “dark circle (Q21)” were higher in the younger group than those in the older group, while logit values for “tinnitus (Q13),” “palpitation (Q14),” “startled by faint noise (Q15),” “joint pain (Q19),” and “itching (Q24)” were higher in the older group than those in the younger group. Therefore, a total of 16 items with DIF by gender or age were removed and nine items, including “breath shortness (Q4),” “stomach fullness (Q6),” “poor appetite (Q7),” “head unclearness (Q10),” “dizziness (Q12),” “chest discomfort (Q16),” “flank pain (Q18),” “lumps (Q22),” and “fatigue (Q25)” were selected for the Rasch analysis.

Table 4 lists the fit levels of the nine questionnaire items. In the first analysis, “lumps (Q22)” showed fitting error (infit = 1.64 and outfit = 1.62). Therefore, the second analysis was conducted after removing “lumps” from the item pool. As a result, eight items except for “lumps” were free of fitting error, showing a range of infit and outfit values from 0.79 to 1.39, and hence, another iteration for fitting analysis was not considered. Among the raw or overall scores for the eight items, “poor appetite (Q22)” was the lowest (score = 697), while “fatigue (Q25)” was the highest (score = 1150), indicating that “fatigue” was the most frequently answered symptom for the subjects with PP.  Table 5 lists the dimensionality results of the 8 items for the Rasch analysis. Unexplained variance in the first contrast was 1.598 (<3.0), implying that the 8-item questionnaire was unidimensional. According to the category response, DIF, fitting, and dimensionality tests of the Rasch analysis, the 8-item PPQ (PPQ-8) rated on a 6-point Likert scale was finally determined.

Table 6 lists the EITC results by three percentile (25%, 50%, and 75%) points. The Rasch analysis suggested the reduction of the 25-item PPQ to eight items; hence, the top three items were extracted from each percentile and summed up to 9 items. While matching the numbers of the EITC items with those of the PPQ-8, “stomach fullness (Q6),” showing the lowest EITC (*r* = 0.453), was removed from the 9 items. Finally, 8 items, including “breath shortness (Q4),” “indigestion (Q5),” “head unclearness (Q10),” “headache (Q11),” “dizziness (Q12),” “palpitation (Q14),” “chest discomfort (Q16),” and “limb heaviness (Q20),” were determined as the 8-item PPQ by EITC. Principal component analysis revealed that the 8-item PPQ by EITC was unidimensional like the PPQ-8 (percentage of variance = 53.637).

The Cronbach's alpha coefficient for the EITC questionnaire was 0.875 and 2.23 for PPQ-8.  Table 7 lists the ROC curve analyses of the 8-item questionnaire extracted from the EITC and Rasch analyses. A previous study reported that the sensitivity, specificity, AUC, and cut-off points of the 25-item PPQ were 83.8%, 83.3%, 0.860 (95% confidence interval: 0.759–0.960), and 5 points, respectively. The AUC levels for the 8-item PPQ using EITC and Rasch analysis were 0.799 (95% confidence interval: 0.668–0.930) and 0.759 (95% confidence interval: 0.620–0.898), respectively. This indicated that the two 8-item questionnaires had moderate accuracy for the determination of the PPQ, similar to the 25-item PPQ. While calculating the maximum Youden index, the sensitivity, specificity, and cut-off points of the 8-item questionnaire were 61.4%, 88.2%, and 28 points, respectively, using ETIC and 70.5%, 76.5%, and 23 points, respectively, for the Rasch analyses. While calculating the minimum Euclidean distance, the sensitivity, specificity, and cut-off points of the 8-item questionnaire were 70.5%, 76.5%, and 25 points, respectively, using EITC, and 70.5%, 76.5%, and 23 points, respectively, for the Rasch analyses.

## 5. Discussion

In this study, a reduced version of the 8 items of the PPQ was developed using Rasch analysis. As EITC analysis has been utilised in some studies to shorten the original questionnaire, another short-form PPQ was developed using EITC analysis, and its results were compared with the results of the PPQ-8, developed through Rasch analysis [14, 18]. Furthermore, the discriminative power of the two versions of the short form of the PPQ was compared with that of the 25-item PPQ using ROC curve analysis. Like most questionnaires developed by classical test theory, the original PPQ version was limited in that it could not present the information of item hierarchy relating to the respondents' ability and item difficulty. Therefore, Rasch analysis was utilised to address concerns regarding the difficulty of items and the ability of the subjects to answer the PPQ.

This study found that among the 7 response categories of the 25-item PPQ, categories 3 (“disagree”) and 4 (“neither disagree nor agree”) were disordered or did not differentiate as predicted. One possibility behind this disordering might be the confusing semantics of category labels [32]. Specifically, participants might have been confused with the neutral response (“neither disagree nor agree”) and slight negative response (“disagree”) among the 7 response categories. After combining the two categories, six response categories satisfied the criteria for the minimum number of each category, outfit MnSq, and step calibration ordering. Moreover, the probability curve showed that the peaks of the six categories did not overlap. Therefore, a 6-point Likert scale, excluding the neutral response, was recommended for future use of the PPQ-8.

The DIF emerged when the heterogeneous groups within the sample responded differently to an item, despite equal levels of the construct that was measured. The DIF analysis compares the logit values of the two groups within a sample. A logit is defined as the natural log of an odds ratio, and greater logits represent increasing item severity [13]. In this study, 16 items were removed from the 25-item PPQ because there were significant differences in the logit values between gender and age. The remaining 9 items were not affected by gender and age, indicating that these 9 items were robust against bias due to the subgroup differences.

The fit analysis found that there were outfit or infit errors for “lumps (Q22).” The outfit is more sensitive to unexpected responses in items that are far from person measure, while the infit is more sensitive to unexpected responses in items that are close to the person measure [33]. The following fit analysis excluding “lumps” showed that the other 8 items were free of fitting errors. Therefore, it appeared that the overall scale of the 8-item PPQ measured something related to the PP without any overestimation or redundancy. From the item response theory point of view, person reliability refers to the differences between high and low respondents and is presented as a separation index. A low separation index indicates the limitation of a questionnaire to assess changes in the underlying trait of an individual [34]. This study showed that the PPQ-8 separation index was 2.23, indicating a satisfactory ability to distinguish between high and low respondents. The 8-item PPQ, according to the EITC analysis, had a “good” internal consistency level (Cronbach's alpha coefficient = 0.875) and was unidimensional, similar to the 8-item PPQ developed via Rasch analysis. Among the 8 items, 4 including “breath shortness (Q4),” “head unclearness (Q10),” “dizziness (Q12),” and “chest discomfort (Q16)” were included in the two versions of the short form PPQ.

In the ROC analysis, the discriminative ability of the 8-item PPQ by EITC (AUC = 0.799) was “moderate,” which was similar to that of the PPQ-8 by Rasch analysis (AUC = 0.759). Considering that the AUC level of the original 25-item PPQ was 0.860, it seemed that the two 8-item PPQs through EITC or Rasch analysis might not have decreased the discriminative ability of the 25-item PPQ. In terms of determination of the cut-off points, the sensitivity levels at the maximum Youden index were lower than the specificity levels for the EITC, indicating an increased possibility of false negativity. Alternatively, the sensitivity levels at the minimum Euclidean distance were similar to the specificity levels, and the cut-off points by the minimum Euclidean distance were lower than those by the maximum Youden index. Therefore, 25 points for the EITC-PPQ, using a minimum Euclidean distance, were recommended. Interestingly, the PPQ-8 by Rasch analysis showed the same sensitivity, specificity, and cut-off points (70.5%, 76.5%, and 23 points, respectively) as the maximum Youden index and minimum Euclidean distance.

However, it should be noted that despite satisfactory reliability and discriminative ability, a limitation of the 8-item PPQ by EITC, that it did not present the information of item hierarchy or DIF characteristics for the subgroups, might remain. Another concern of the 8-item PPQ by EITC was that the determination of the item numbers of the PPQ was somewhat arbitrary because the item numbers in the EITC analysis were forced to match those in the Rasch analysis. Therefore, this study suggested that PPQ-8 by Rasch analysis might be preferable to EITC for future use to evaluate PP.

It should also be noted that this study did not include an examination of the content validity of the short-form PPQ. Previously, the content validity of the pilot version of the PPQ was examined, where 17 clinicians were asked to rate the importance of each questionnaire item for the PP, using a 7-point scale [35]. The clinical importance of “sputum” for the PP was top-ranked (6.4 points), and the importance of “sickness (6.2 points),” “feeling of foreign body (5.9 points),” “dizziness (5.7 points),” and “dark circle (5.6 points)” followed in the study. Additionally, the reduced items via the EITC and Rasch analyses were not related to the rank of clinical importance for the pilot version of the PPQ. Considering that the 25-item PPQ was developed from the items that were rated only on at least 4 points of clinical importance by clinicians and the PPQ-8 items were reduced from those of the 25-item PPQ, it appears that satisfactory content validity of the 25-item PPQ may guarantee the content validity of the 8-item PPQ.

## 6. Limitations

This study had some limitations. Although Rasch analysis presented information on DIF, it was affected by sample characteristics, such as environmental and racial differences. Therefore, item reduction of the original PPQ had to be performed in the other population using Rasch analysis. In this study, item reduction was conducted for normal participants, whereas ROC analysis was conducted for inpatients. Therefore, the differences between the two samples may have affected the results of the ROC curve analysis. Further studies are needed to overcome these limitations regarding the environmental and racial differences and the sample characteristics.

## 7. Conclusion

In this study, the short-form PPQ was developed using Rasch analysis based on retrospective data from 291 normal participants and 61 inpatients. Together with Rasch analysis, another short-form PPQ was developed using EITC analysis, and the results of the 2 short-form PPQs and the original version of the PPQ were compared. The Rasch analysis results suggested a 6-point response category for the PPQ and finally determined the PPQ-8 consisting of eight items, free of fitting errors or DIF variability. Furthermore, the PPQ-8 had satisfactory reliability, concurrent validity, unidimensionality, fitting levels, sensitivity, and specificity, as well as the moderate discriminative ability of PP. Despite the 8-item PPQ using EITC analysis showed similar levels of reliability, validity, and discriminative ability of PP to those of the PPQ-8, it could not present the information of item hierarchy and DIF. In conclusion, the PPQ-8 by Rasch analysis was recommended for future use to evaluate the clinical severity of PP, reduce the response burden, and minimise differences between gender and age.

## Figures and Tables

**Figure 1:** Probability curves of the 7-point (a) and 6-point (b) responses. C1 (category 1), disagree very strongly; C2 (category 2), disagree strongly; C3 (category 3), disagree; C4 (category 4), neither disagree nor agree; C5 (category 5), agree; C6 (category 6), agree strongly; and C7 (category 7), agree very strongly. The arrow indicates the peak of the C4 curve in 1B.

**Table 1:** The 25-item phlegm pattern questionnaire.

No.	Item	Condition
Q1	I have a cough	Cough
Q2	I have sputum in my throat	Sputum
Q3	I feel a foreign body present in the throat, neither swallowed nor ejected	Feeling of a foreign body
Q4	I feel shortness of breath	Breath shortness
Q5	I have indigestion	Indigestion
Q6	I have a feeling of fullness with minimal food intake	Stomach fullness
Q7	I have a poor appetite	Poor appetite
Q8	My stomach or intestine rumbles	Abdominal rumbling
Q9	I feel sick to the stomach	Sickness
Q10	I feel unclear in the head	Head unclearness
Q11	I have a headache	Headache
Q12	I feel dizzy	Dizziness
Q13	I have ringing in my ears	Tinnitus
Q14	I feel my heart palpitating	Palpitation
Q15	I am startled by faint noise	Startled by faint noise
Q16	I feel heavy in the chest	Chest discomfort
Q17	My stool is mucousy	Mucousy stool
Q18	I have flank pain	Flank pain
Q19	I have pain in the joints	Joint pain
Q20	I feel heavy or weak in the limbs	Limb heaviness
Q21	I have dark circles under my eyes	Dark circle
Q22	I have a lump in my body	Lumps
Q23	My face is yellowish	Yellow face
Q24	I feel itchy	Itching
Q25	I feel fatigued	Fatigue

**Table 2:** Category characteristics of the 7- and 6-point Likert scales.

Scale	Category (response)	Observed count (%)	Average measure	Expected measure	Infit MnSq	Outfit MnSq	Step calibration	Category measure
7-point Likert	1 (disagree very strongly)	829 (11)	−1.39	−1.24	0.86	0.93	None	−3.06
	2 (disagree strongly)	2276 (31)	−0.57	−0.63	0.99	0.94	−1.89	−1.21
	3 (disagree)	873 (12)	−0.34	−0.37	0.96	1.06	0.47	−0.44
	4 (neither disagree nor agree)	1290 (18)	−0.15	−0.16	0.97	1.20	−0.65^*∗*^	0.03
	5 (agree)	1093 (15)	0.01	0.03	1.06	1.24	0.10	0.52
	6 (agree strongly)	677 (9)	0.16	0.22	1.13	1.27	0.60	1.29
	7 (agree very strongly)	237 (3)	0.46	0.42	1.01	1.26	1.37	2.74

6-point Likert	1 (disagree very strongly)	829 (11)	−1.78	−1.65	0.91	0.93	None	−3.37
	2 (disagree strongly)	2276 (31)	−0.72	−0.77	0.94	0.89	−2.14	−1.46
	3 (disagree)	2163 (30)	−0.31	−0.34	0.97	1.10	−0.49	−0.23
	4 (agree)	1093 (15)	−0.02	−0.01	1.02	1.12	0.51	0.56
	5 (agree strongly)	677 (9)	0.22	0.30	1.11	1.22	0.62	1.41
	6 (agree very strongly)	237 (3)	0.61	0.61	1.04	1.24	1.50	2.85

^*∗*^Disordering response category, where the step calibration value became lower than that of the previous category.

**Table 3:** Differential item functioning results by gender and age.

Item	Gender				Age			
	Male (logit)	Female (logit)	Chi-square value	*P* value	Younger (logit)	Older (logit)	Chi-square value	*P* value
Cough (Q1)	0.12	−0.10	4.753	**0.029**	<0.01	<0.01	1.631	0.202
Sputum (Q2)	0.39	−0.32	24.105	**<0.001**	0.14	−0.13	8.021	**0.005**
Feeling of foreign body (Q3)	0.19	−0.16	3.677	0.055	0.11	−0.11	4.595	**0.032**
Breath shortness (Q4)	0.06	−0.06	1.678	0.195	−0.03	0.03	0.006	0.937
Indigestion (Q5)	−0.06	0.05	1.502	0.220	0.15	−0.15	4.501	**0.034**
Stomach fullness (Q6)	−0.04	0.03	0.297	0.586	−0.03	0.03	0.070	0.790
Poor appetite (Q7)	−0.07	0.05	2.314	0.128	0.01	−0.01	0.031	0.861
Abdominal rumbling (Q8)	0.27	−0.23	8.709	**0.003**	0.21	−0.21	7.224	**0.007**
Sickness (Q9)	−0.02	0.02	0.620	0.431	0.10	−0.10	4.556	**0.033**
Head unclearness (Q10)	0.10	−0.08	2.587	0.108	0.09	−0.08	1.980	0.159
Headache (Q11)	−0.06	0.05	0.038	0.846	0.12	−0.12	4.209	**0.040**
Dizziness (Q12)	−0.12	0.10	0.122	0.727	0.07	−0.07	2.535	0.111
Tinnitus (Q13)	0.07	−0.06	0.148	0.701	−0.18	0.17	9.853	**0.002**
Palpitation (Q14)	−0.24	0.20	8.885	**0.003**	−0.15	0.14	5.061	**0.025**
Startled by faint noise (Q15)	−0.36	0.29	19.496	**<0.001**	−0.15	0.14	5.374	**0.020**
Chest discomfort (Q16)	−0.13	0.10	1.362	0.243	−0.09	0.09	2.642	0.104
Mucousy stool (Q17)	0.15	−0.13	4.981	**0.026**	0.93	−0.03	<0.001	0.999
Flank pain (Q18)	-0.01	0.00	0.071	0.790	−0.09	0.09	0.988	0.320
Joint pain (Q19)	−0.22	0.18	7.847	**0.005**	−0.40	0.38	21.922	**<0.001**
Limb heaviness (Q20)	−0.17	0.14	4.309	**0.038**	−0.09	0.09	2.550	0.110
Dark circle (Q21)	−0.01	0.01	1.003	0.317	0.32	−0.31	17.714	**<0.001**
Lumps (Q22)	0.08	−0.07	1.439	0.230	−0.09	0.08	3.284	0.070
Yellow face (Q23)	−0.19	0.16	8.885	**0.003**	−0.04	0.04	1.679	0.195
Itching (Q24)	0.29	−0.24	9.435	**0.002**	−0.08	0.08	3.955	**0.047**
Fatigue (Q25)	−0.04	0.04	0.840	0.360	0.09	−0.08	0.517	0.473

The *P* values in bold indicate significant differences in logit values between gender and age.

**Table 4:** Item difficulty and fitting levels of the short form PPQ using Rasch analysis.

Iteration	Item	Raw score	Model measure	Infit MnSq	Outfit MnSq
First	Lumps (Q22)	654	0.88	1.64	1.62
	Flank pain (Q18)	702	0.60	1.30	1.27
	Poor appetite (Q7)	697	0.63	1.18	1.13
	Fatigue (Q25)	1150	−1.34	1.01	1.05
	Stomach fullness (Q6)	820	<0.01	1.00	1.03
	Dizziness (Q12)	911	−0.40	0.84	0.87
	Head unclearness (Q10)	965	−0.62	0.80	0.81
	Chest discomfort (Q16)	847	−0.12	0.76	0.76
	Breath shortness (Q4)	745	0.37	0.74	0.75

Second	Flank pain (Q18)	702	0.77	1.39	1.34
	Poor appetite (Q7)	697	0.80	1.23	1.17
	Stomach fullness (Q6)	820	0.12	1.07	1.08
	Fatigue (Q25)	1150	−1.35	1.04	1.07
	Dizziness (Q12)	911	−0.31	0.92	0.93
	Head unclearness (Q10)	965	−0.56	0.86	0.87
	Chest discomfort (Q16)	847	−0.01	0.81	0.81
	Breath shortness (Q4)	745	0.52	0.80	0.79

**Table 5:** Dimensionality results of the 8-item Rasch analysis.

Standardised residual variance	Eigenvalue (%)
Total raw variance in observations	17.339 (100)
Raw variance explained by measures	9.339 (53.9)
Raw variance explained by persons	3.724 (21.5)
Raw Variance explained by items	5.616 (32.4)
Raw unexplained variance (total)	8.000 (46.1)
Unexplained variance in 1^st^ contrast	**1.598** (9.2)
Unexplained variance in 2^nd^ contrast	1.511 (8.7)
Unexplained variance in 3^rd^ contrast	1.169 (6.7)
Unexplained variance in 4^th^ contrast	1.070 (6.2)
Unexplained variance in 5^th^ contrast	0.991 (5.7)

The value in bold indicates an acceptable eigenvalue of the variance for unidimensionality (<**2.0**).

**Table 6:** Equidiscriminative item-total correlation (EITC) results by three percentile points.

25% cut-off points of the total scores (86 points)	Spearman correlation	50% cut-off points of the total scores (99 points)	Spearman correlation	75% cut-off points of the total scores (116 points)	Spearman correlation
**Chest discomfort**	0.553	Dizziness	0.621	Breath shortness	0.556
**Head unclearness**	0.527	**Limb heaviness**	0.565	Dizziness	0.544
**Dizziness**	0.517	Head unclearness	0.560	Chest discomfort	0.522
Breath shortness	0.514	**Breath shortness**	0.558	Palpitation	0.500
Palpitation	0.510	Chest discomfort	0.553	**Headache**	0.493
Headache	0.495	**Palpitation**	0.549	Limb heaviness	0.489
Limb heaviness	0.488	Abdominal fullness	0.547	**Indigestion**	0.471
Indigestion	0.453	Headache	0.526	Head unclearness	0.454
Fatigue	0.447	Sickness	0.518	**Abdominal fullness** ^**a**^	0.453
Abdominal fullness	0.437	Indigestion	0.514	Startled by faint noise	0.451
Cough	0.426	Startled by faint noise	0.496	Sickness	0.441
Startled by faint noise	0.419	Fatigue	0.47^*∗*^	Fatigue	0.418
Tinnitus	0.391	Poor appetite	0.425	Joint pain	0.357
Poor appetite	0.383	Cough	0.404	Cough	0.354
Sickness	0.375	Mucousy stool	0.401	Feeling of foreign body	0.335
Rumbling abdomen	0.373	Flank pain	0.400	Yellow face	0.322
Flank pain	0.371	Feeling of foreign body	0.381	Rumbling abdomen	0.317
Lumps	0.370	Joint pain	0.370	Itching	0.315
Mucousy stool	0.359	Tinnitus	0.364	Mucousy stool	0.313
Sputum	0.351	Rumbling abdomen	0.362	Poor appetite	0.312
Joint pain	0.350	Yellow face	0.357	Flank pain	0.305
Itching	0.350	Sputum	0.352	Tinnitus	0.263
Dark circle	0.326	Itching	0.349	Sputum	0.240
Feeling of foreign body	0.319	Lumps	0.320	Dark circle	0.225
Yellow face	0.316	Dark circle	0.305	Lumps	0.222

Items in bold indicate the top-three questionnaire items, by the three percentile points. ^a^Discarded questionnaire item to match the numbers of questionnaire items by EITC with those by Rasch analysis. All correlations had *P* < 0.01.

**Table 7:** Receiver operating characteristic (ROC) curve analyses of the EITC and the Rasch models.

The 8-item questionnaire by EITC	The 8-item questionnaire by Rasch analysis								
Points	Sensitivity	Specificity	Youden index	Euclidean distance	Points	Sensitivity	Specificity	Youden index	Euclidean distance
18.5	0.886	0.471	0.357	0.541	15.5	0.909	0.353	0.262	0.653
19.5	0.864	0.471	0.335	0.546	16.5	0.909	0.412	0.321	0.595
20.5	0.818	0.471	0.289	0.559	17.5	0.864	0.412	0.275	0.604
21.9	0.773	0.588	0.361	0.470	18.5	0.841	0.471	0.311	0.553
22.5	0.727	0.706	0.433	0.401	19.5	0.795	0.529	0.325	0.513
23.5	0.705	0.706	0.411	0.416	20.5	0.727	0.588	0.316	0.494
24.5	0.705	0.765	0.470	**0.377**	21.5	0.727	0.647	0.374	0.446
25.5	0.659	0.824	0.483	0.384	22.5	0.705	0.765	**0.469**	**0.378**
26.5	0.636	0.824	0.460	0.404	23.5	0.636	0.765	0.401	0.433
27.5	0.614	0.882	**0.496**	0.404	24.5	0.500	0.824	0.324	0.530
28.4	0.591	0.882	0.473	0.426	25.5	0.432	0.824	0.255	0.595
28.9	0.568	0.882	0.450	0.448	26.5	0.409	0.882	0.291	0.603
29.5	0.409	0.882	0.291	0.603	27.5	0.341	0.882	0.223	0.670
31.0	0.341	0.882	0.223	0.669	28.5	0.273	0.882	0.155	0.737
32.5	0.318	0.882	0.200	0.692	29.5	0.205	0.882	0.087	0.804

The values in bold indicate the maximum Youden index and minimum Euclidean distance obtained using ROC curve analyses.

## Data Availability

The data used to support the findings of this study have not been made available because the data contain personal information.
